This article has been retracted.

# Analysis of Signs and Effects of Surgical Breast Cancer Patients Based on Big Data Technology

**DOI:** 10.1155/2022/3373553

**Published:** 2022-09-23

**Authors:** Zhen Hong, Qin Xu, Xin Yan, Ran Zhang, Yuanfang Ren, Qian Tong

**Affiliations:** ^1^School of Nursing, Jiangsu Jiankang Vocational College, Nanjing 211800, China; ^2^School of Nursing, Nanjing Medical University, Nanjing 211166, China; ^3^Department of Thyroid and Breast Surgery, The First Affiliated Hospital of Nanjing Medical University, Nanjing 210029, China

## Abstract

Big data in health care has gained popularity in recent years for disease prediction. Breast cancer infections are the most common cancer in urban Indian women, as well as women internationally, and are impacted by many events across countries and regions. Breast malignant growth is a notable disease among Indian women. According to the WHO, it represents 14% of all malignant growth tumors in women. A couple of studies have been directed utilizing big data to foresee breast malignant growth. Big data is causing a transformation in healthcare, with better and more ideal results. Monstrous volumes of patient-level data are created by using EHR (Electronic Health Record) systems data because of fast mechanical upgrades. Big data applications in the healthcare business will assist with improving results. Conventional forecast models, then again, are less productive in terms of accuracy and error rate because the exact pace of a specific calculation relies upon different factors such as execution structure, datasets (little or enormous), and kinds of datasets utilized (trait-based or picture based). This audit article looks at complex information mining, AI, and profound learning models utilized for recognizing breast malignant growth. Since “early identification is the way to avoidance in any malignant growth,” the motivation behind this audit article is to support the choice of fitting breast disease expectation calculations, explicitly in the big information climate, to convey powerful and productive results. This survey article analyzes the precision paces of perplexing information mining, AI, and profound learning models utilized for distinguishing breast disease on the grounds that the exactness pace of a specific calculation relies upon different factors such as execution structure, datasets (little or enormous), and dataset types (quality based or picture based). The reason for this audit article is to aid the determination of suitable breast disease expectation calculations, explicitly in the big information climate, to convey successful and productive outcomes. Thus, “Early discovery is the way to counteraction in the event of any malignant growth.”

## 1. Introduction

Big data has its roots from 1941 when the Oxford dictionary of English published the first mention to the concept of “information explosion.” In a study published by the National Academy of Sciences in 1996, James Maar emphasized the concept of a “huge data set” (1). However, it was not until 1997 that the term “Big Data” was coined in an article in the Association for Computing Machinery's Digital Library (2), alluding to the technological issue of interpreting massive volumes of data. Since then, it has been used to refer to “structured or unstructured data whose extremely huge volume necessitates specialised analysis techniques.” Over the last decade, internet behemoths (Google, Amazon, Facebook, Apple, and Twitter) have built such technologies, ensuring a consistent marginal cost of data exploitation regardless of scale.

Today, Big Data is defined by the 5 vs of the data exploited: volume, velocity, variety, veracity, and value. The vast volumes and fast speed of data processing are the results of lower storage prices and increased computing capability [1]. The rising digitization of information media has resulted in a greater diversity of data (pictures, texts, databases, connected devices, and so on). Finally, the accuracy of the data, which determines the job's worth, is an important consideration for any automated data analysis project [2–5].Indeed, if the data is huge, precise, and well-suited to the problem at hand, an algorithm can be tremendously strong. Multiplying sources and crossings without concern for data quality may result in incorrect results, particularly in the health area. The rise of “Open Data,” which refers to data gathered and kept by multiple organizations and made available to individuals and businesses, has coincided with the rise of the internet development of big data [6].

The 5 vs, on the other hand, are insufficient to capture the core of big data's innovation. The knowledge of these algorithms is at the core of data scientists' work.

Breast cancer diagnosis and treatment have come a long way in the previous three decades. Individual or organized breast screening activities, as well as advances in breast imaging equipment, have all contributed to this breakthrough. Without a doubt, a sub-space of man-made consciousness known as “AI” permits designers to make algorithms equipped for collecting information and knowledge from tests without being directed by people or expressly modified to deal with a particular errand, bringing about their focal job in the data esteem chain, with the rest of to propels in careful methods or clinical medicines [7–11].

The advent of big data technology has recently piqued the curiosity of medical professionals concerned with breast health. Indeed, storage capacity has expanded significantly over the previous three decades, bringing about larger amounts and a more noteworthy variety of clinical information that has been saved (mammography filters, 3D ultrasound, MRI, genomic information, neurotic information, and so forth). As of not long ago, this information was every now and again utilized at a singular level over the course of time to produce a conclusion and a helpful arrangement, follow ailment improvement, and conjecture a patient's forecast. Besides, just coordinated information on a factual scale was utilized, which addressed just a tiny level of the open and useable data sources.

The rest of putting away information cemeteries was scarcely apparent to clinical professionals. The primary guarantee of great data is that it will empower the utilization of all information sources, even unstructured ones such as text-based patient reports or photographs, influencing clinical exploration and, at last, patient consideration [12, 13].

To completely appreciate how big data might improve breast health care, two developments must be examined. To start, the production environment that has arisen throughout the past ten years takes into account the execution of predefined procedures on immense volumes and various kinds of data. Second, AI algorithms and their programming language executions might gain from data to reveal examples and correlations, coming about in significant insights. Data researchers are seasoned veterans at dealing with these unique techniques [14].

The success of these cutting-edge investigations is dependent on transdisciplinarity. It takes time to develop a shared semantics between medical personnel and data scientists, and the breast disease units' experience working in transversal organizations will be invaluable in developing a framework for these interactions. Patients and, more broadly, civic society should be included in Big Data projects, in addition to medical professionals and data scientists, because only rigorous adherence to privacy standards can ensure their success and profitability [15, 16].

### 1.1. Breast Cancer

Breast disease is a fiery growth that begins in the breast and spread to the remainder of the body. Disease emerges when cells start to multiply wildly. Breast malignant growth is a gathering of infections wherein breast tissue cells move and create uncontrolled, finishing in a protuberance or mass. Most breast tumors start in the dairy organs. Mammograms, breast self-assessment (BSE), biopsy, and refined breast tissue measurements are used to assess breast malignant growth. A medical operation, radiation, chemical treatment, chemotherapy, and laser treatment can all be used to treat breast cancer.

At the point when harmful development cells enter the circulatory or lymphatic frameworks and travel to various pieces of the body, breast ailment could spread. Breast cancerous growth cells typically structure an irregularity or cancer, which should be visible on an X-beam or felt as a firm mass. Monitoring controllable gamble variables can assist with lessening the probability of creating breast malignant growth [17]. Breast malignant growth is principally a female infection, but it is turning out to be more normal in men.

#### 1.1.1. Types of Breast Cancer

Obtrusive breast cancer and noninvasive breast cancer are two kinds of breast diseases that can be characterized based on regardless of whether the malignant growth has spread (Figure 1) [18].

Obtrusive breast disease, then again any sort of breast-threatening development that has spread to the breast tissues, is suggested as nosy ductal carcinoma (IDC) which attacks the incorporating tissues in the breasts, making them substantial and perceptible on mammograms. Intrusive breast disease represents 81% of all cases of invasive breast disease. Then again, any sort of dangerous breast development that has spread to the incorporating breast tissues is implied as meddlesome ductal carcinoma (IDC) attacks the including tissues of the breasts, making them discernible and perceptible on mammograms. Obtrusive breast malignant growth represents 81% of all cases. Invasive lobular carcinoma (ILC) infiltrates the breast tissues on both sides and is microscopically identified as inflammatory carcinoma, often known as IBC (fiery breast disease); it is an intriguing and perilous sort of breast malignant growth that appears as a rash or bothered skin region [19, 20].

It blocks the lymph vessels in the skin of the breasts. Since searing breast disease cannot be perceived by mammography or ultrasound, it ought to be found imperceptibly [21–24]. Paget's infection is an especially interesting sort of breast disease. Paget's disease of the breast starts on the areola and spreads to the encompassing dark circle of skin (areola). Intrusive ductal carcinoma is the medical term for male breast cancer in cutting-edge stages, Figure 2.

#### 1.1.2. Breast Cancer Symptoms and Signs

Another lymph center point or hard mass around the Breast or underarm district is a truly common breast-threatening development sign. Breast dangerous development is consistently portrayed by a simple, hard knot with sporadic edges; however, it can likewise be a delicate, delicate mass. Breast malignant growth frequently has no side effects in light of the fact that the cancer is little and simple to treat. Consequently, screening is vital for right on-time identification. The signs and symptoms of breast cancer vary from person to person. Some folks do not have any symptoms or signs at all [17].

#### 1.1.3. Breast Cancer Stages and Survival Rate

Cells in the conduit lining or a segment of the breast are strange, as indicated by the SEER Committee's stage framework (surveillance, epidemiology, and end results). Breast disease is bound to create in one or the two breasts. At this moment, the perseverance rate is 100%. Breast disease is a sort of harmful development that impacts the tissues of the breast. The disease is short of one inch in broadness [25–27]. This stage has a 95% to 98 percent chance of perseverance. It has something to do with breast tissues, also. Growth is more modest than two crawls in measurement. The illness is malignant growth and may grow to the assistant lymph hubs. The endurance rate is currently at 88 percent breast tissues are affected. The tumor is more than two creeps in breadth. The disease might expand to the assistant lymph hubs. These things could occur as irritation, dimpling, or an adjustment of skin cooler. Right now, the endurance rate is somewhere close to half and 60%. Notwithstanding the breast, the disease has spread to different pieces of the body. Right now, the opportunity for endurance ranges somewhere in the range of 15% – 20%.

#### 1.1.4. Breast Cancer Causes

The progression or change in the DNA of the cells is the reason for this. A percentage of the danger factors are benign conditions, such as hyperplasia, which raise the risk of breast cancer. Having a history of malignant development increases your chances of creating disease [6].

### 1.2. Breast Cancer: Types, Statistics and Tооls for Early Detection

#### 1.2.1. Breаst Cancer Types and Statistics

Breast malignant growth creates when cells in the breast start to multiply wildly. These cells generally combine to make cancer, which should be visible on an x-beam or as a felt knot. If the cells of the growth penetrate (attack) surrounding tissues or spread (metastasize) to other parts of the body, the cancer is dangerous (carcinogenic). Breast disease fundamentally influences ladies; however, it can likewise affect men. Breast disease can start in various areas of the Breast. By far, most breast tumors start in the pipes that convey milk to the areola (malignant ductal growths). A few malignancies (lоbular growths) begin in the organs that make breast milk [14, 28].

It is basic to comprehend that by far, most breast knots are not threatening; all things being equal, they are harmless. Harmless breast cancers are harmless developments that do not spread outside of the breast and do not imperil one's life. Some harmless breast knots, then again, can build a lady's gamble of creating breast disease. A medical services expert ought to assess any bump or change in the breast to decide if it is harmless or dangerous and whether it might adjust future disease risk. Breast disease can possibly spread to different pieces of the body through the lymphatic framework [15].

The lymph framework is made up of y lymph centers, lymph chambers, and lymph liquids that can be tracked down all through the body [29–31]. Lymph centers are little bean-molded groups of resistant framework cells connected together by lymph (or lymphatic) veins. Lymph vessels are like little veins in that they transport lymph (as opposed to blood) out from the breast. Lymph contains both tissue liquids and waste, as well as insusceptible compromised framework cells. Breast disease cells are fit for entering lymphatic channels and topping off lymph hubs [18].

There is a chance that cancerous growth cells have spread to your lymph nodes, and a huge likelihood they have spread to different spots of your body (metastasized). Early location is basic for human existence, particularly on account of forceful breast malignant growth. Breast malignant growth is the most regular sickness among ladies around the world, as indicated by the World *Cancer* Research Fund International (WCRFI), with over 1.7 million new cases recognized in 2012. It is the second most normal disease on the planet [20, 32–34]. These record for around 12% of all new disease cases and 25% of all malignant growth cases in ladies.

Age standardized rate per 1, 00,000 (world).

## 2. Review of the Literature

Many studies on breast cancer in the field of medical data analysis have been distributed, and most of them guarantee to have extraordinary grouping exactness.

An assessment report has been distributed in which they characterized breast disease threatening development involving numerous techniques, including choice, highlight extraction, and component gathering strategies. The WEKA procedure is used to break down breast malignant growth illness data from the UCI store, and the portrayed strategies are utilized to arrange details exactly. This study demonstrates unequivocally that the information-gathering technique is efficient in predicting breast cancer sickness. The WEKA device is highly considered in data mining as one of the most effective and dependable data classification strategies. SVM outperformed other methods on the data set for breast cancer malignant development and produces consistent results. With an accuracy rate of 82.53 percent, 286 instances and 10 characteristics of breast cancer disease were investigated.

The authors of [6]fostered a framework plan for foreseeing the event of breast disease threatening development in the beginning phases by assessing the littlest assortment of factors from the clinical dataset. The Wisconsin breast malignant growth dataset (WBCD) was used to carry out the suggested investigation. The capacity of the proposed technique is determined by comparing actual with expected features and obtaining characterisation exactness. The results suggest that this inquiry has the highest categorization accuracy of 99.28%.

“Addresses the execution of a progress improvement algorithm to mine two distinctive datasets in AI using four unique progression smoothing techniques.” Iris Data We used the set and the breast cancer dataset as informational data. A set to test the selected suggested improvement estimates [15].

The cerebrum affiliation (NN) is used in the solicitation issue of this exploration, close by four streamlined upgrade strategies: whale optimization algorithm (WOA), dragonfly algorithm (DA), multiverse optimization (MVA), gray wolf optimization (GWO). For precise choices of the proposed enhancement processes, an assortment of control limits was analyzed. Concerning intermingling, runtime, characterisation rate, and MSE, the comparison study shows that the GWO and MVO outperform both the WO and the DA. Hybrid algorithms that combine two different optimization methodologies could be investigated further in the future for data mining tasks” [20].

Recognized five managed AI computations are support vector machine (SVM), K-nearest neighbor method, random forest, artificial neural network (ANN), and logistic regression (LR) [1]. The UCI Storage House contains associations with the Wisconsin Breast Cancer Observation Dataset. Accuracy, mindfulness, specificity, accuracy, negative predictable values, false negative rates, interesting positive rates, *F*1 scores, and Matthews correlation coefficients are fully used to examine experimental results. The accuracy and accuracy of the ANN is only 98.57%, 97.82%, and 0.9890, which are the highest, while the accuracy and accuracy of the SVM are the second highest, with *F*1 scores of 97.14%, 97, 14%, and .9890, respectively.

“Working on the performance of most grouping algorithms by applying techniques for highlight choice to limit how much elements” [20]. Certain properties are more important than others and affect the results of order calculations. The inspiration that drives this study is an overview of the accuracy of some recent information mining estimates in predicting the recurrence of breast disease. It utilizes molecule swarm advancement as a component choice in three notable classifiers: Naive Bayes, K-closest neighbor, and quick choice tree student to move along the prediction model's accuracy. The performance of naive Bayes was superior with and without PSO (particle swarm optimization), but when combined with PSO, the other two approaches improved.”

Support vector machine (SVM)-based BCD model for distinguishing breast disease with 10-overlap cross approval. At the point when there are numerous information highlights for malignant growth ID, the undertaking gets more troublesome [15]. Principal component analysis (PCA) is a procedure for restricting the element region extending from a higher to a lower aspect. The PCA refines the model's accuracy based on the assessment results. Other learning calculations such as decision tree (DT), random forest, k-nearest neighbor method (k-NN), stochastic gradient descent (SGD), AdaBoost, neural network (NN), and naave Bayes have been proposed. It is displayed in a different way. BCD model. (query)According to the *F*1 measure, ROC twist, accuracy, lift curve, and calibration chart, the proposed BCD model provides excellent accuracy among the various model strategies investigated. The proposed BCD model has the most elevated AUC of 0.995 and the most noteworthy precision of 98.1 percent among different models tried.”

The effectiveness of the five nonlinear machine learning methods is A.A. Evaluated in an 18-inch study by Bataineh: Multilayer Perceptron (MLP), K-nearest neighbor method (KNN), classification and regression tree (CART), Gaussian Naive Bayes (NB), and support vector machine (SVM) [37, 38] when it comes to data classification, the main goal is to evaluate the performance and feasibility of each algorithm in terms of accuracy, accuracy, and validation of characteristic tests. MLP has 96.70% accuracy when compiling data. This is more obvious than the other four algorithms. After evaluation, the accuracy and validation of the predictive model are evaluated by using the K-overlap mutual recognition method for ambiguous data. According to the results of this review, the accuracy, accuracy, and validation of the MLP model were highest at 99.12 percent, 99.00 percent, and 99.00 percent, respectively. The review relied on the Wisconsin Breast Cancer Diagnosis (WBCD) dataset.

Jing Zheng, Denan Lin, ZhongjunGao, Shuang Wang, Mingjie He, Jipeng Fan, Jing Zheng, Denan Lin Den Mathematically proposed an efficient AdaBoost algorithm for deep learning support to identify harmful enhancements to the breast (DLA-EABA) was run by using the current PC-development carried out. Notwithstanding customary PC vision methodologies, deep convolutional neural networks are being used to investigate tumour classification methods that use transfers (CNNs). This examination centers around deciding the best strategy by consolidating a few methodologies for choosing and separating highlights, as well as assessing their result utilizing grouping and division algorithms, which are essential for AI techniques. The preliminary results exhibit a serious level of precision of 97.2 percent, responsiveness of 98.3 percent, and particularity of 96.5 percent when contrasted with other contemporary systems.”

## 3. Research Methodology

Pertinent distributions for this audit were found via looking through Google Scholar, Research Gate, PubMed, Science Direct, IEEE, and Springer for terms like [“Breast *Cancer*” or “Dangerous development Detection”] + “Man-made intelligence” + [“SVM or ANN”] + [Biosensors or FET or Electrochemical”] [36, 37]. This audit takes care of every one of the applications where breast malignant growth recognition can be applied. Prior to 2018, studies were deemed less relevant because the approaches offered were less accurate, were more expensive, and had a smaller scope of implementation.

## 4. Data Analysis

Zheng, Jing, Lin, Denan, Gao, Zhongjun, Wang, Shuang, He, Mingjie und Fan, Jipeng Entwicklungen *Cancer* arrangement techniques that include moves, notwithstanding conventional PC vision strategies, are as of now being investigated utilizing profound convolutional brain organizations (CNNs). This exploration centers around deciding the ideal strategy by consolidating a few AI procedures with techniques for choosing and removing highlights, as well as assessing their result utilizing order and division calculations. When contrasted with other existing frameworks, the trial results show that the high exactness level of 97.2 percent, awareness of 98.3 percent, and particularity of 96.5 percent are superior.

### 4.1. A Comparative Analysis of Breast Cancer Prediction Techniques (Year 2016 to 2020)

Further study gives a point-by-point portrayal of breast malignant growth grouping utilizing different AI, information mining, and profound learning procedures in light of the Algorithm/technique utilized for expectation, instruments, informational index, information type, and number qualities considered for the review, as displayed in Table 1.

## 5. Result Analysis

We searched the information databases of BMC Bioinformatics, Biomed, Google Scholar, IEEE, Science-Direct, Springer, and Web of Science for the penetration rate and research of huge learning systems in the fields of information mining, AI, and clinical information evaluation. Multiview-Mammography-based informative placement/numerical property-based informative combinations were found to have been used in the evaluation study [39–41]. This genuine Figure 3 and close to assessment Table 1 further shows that mammograms/pictures are used in relatively few examinations of breast-threatening development assumptions. The accessibility of datasets is a critical obstacle to utilizing AI and profound learning strategies to foresee breast malignant growth on the grounds that every strategy requires a lot of preparing information for computational evaluations. We present an outline of information mining, AI, and profound learning approaches in this work, with an accentuation on the precision speed of breast infection assumption. We searched the information databases of BMC Bioinformatics, Biomed, Google Scholar, IEEE, Science-Direct, Springer, and Web of Science for the penetration rate and research of huge learning systems in the fields of information mining, AI, and clinical information evaluation. Multiview-Mammography-based informative placement/numerical property-based informative combinations were found to have been used in the evaluation study [37].

## 6. Conclusion

The basic role of this research article is to identify existing AI and important learning studies that assume the development of harmful breasts and identify the best framework for assessing their proportion. It has been perceived that more work still needs to be carried out from here on out since large information is creating an unrest in medical care at this moment [42, 43].

There is a need to deal with this enormous measure of information since the present advanced medical services require astute incorporation and collection of accessible patient data and PC information, coordinated, semi-organized, and unstructured, in their unique organizations. Second, because of the shortage of accessible datasets, not very many exploration studies on breast disease pictures are led. Accordingly, a model for foreseeing breast malignant growth from a histopathological picture put together informational collections with respect to big information can be proposed. To start, Hadoop engineering can be made to hold information tests to imagine the work on Big information, and afterward, an effective convolutional brain network calculation can be developed for expectation [18].

## Figures and Tables

**Figure 1:** Classification of breast cancer.

**Figure 2:** Preventing breast Cancer stats аccоrding WCRFI [20].

**Figure 3:** Statistical comparison of data mining, machine learning, and deep learning methods for breast cancer prediction over the last 5 years (2016–2020).

**Table 1:** Comparison of breast cancer data mining, machine learning, predictive deep learning techniques [19].

S. no	Author name	Method	Tools	Dataset	Data type	No. of attribute	Performance
1.	Venkateshwara Rao, Mary Gladence	Classification techniques SVM, Naïve Bayes	Weka	UCI machine learning	Numeric attributes	296	Higher accuracy 85%
2.	Madhu kumara, Vijhendra Singh	Classification supervised machine learning algorithm	MAtlab	Wisconsin breast cancer	Numeric	700	KNN classifier with 100%

## Data Availability

The data used to support the findings of this study are included within the article.

## References

[1] Islam M., RezwanulHaque M. d., HasibIqbal, MunirulHasan M. d., MahmudulHasan M. N (2020). Breast Cancer Prediction: A comparative study using machine learning techniques. *SN COMPUTERS SCIENCE*.

[2] Eltalhi S., Kutrani H. (2019). Breast cancer diagnosis and prediction using machine learning and data mining techniques: a review. *IOSR J. Dental Med. Science*.

[3] Ganggayah M. D., Taib N. A., Har Y. C., Lio P., Dhillon S. K. (2019). ‘Predicting factors for survival of breast cancer patients using machine learning techniques. *BMC Medical Informatics and Decision Making*.

[4] Ibrahim A. A., Hashad A. I., Shawky N. E. M. (2017). ‘A comparison of open source data mining tools for breast cancer classification. *Handbook of Research on Machine Learning Innovations and Trends*.

[5] Hosni M., Abnane I., Idri A., de Gea J. M. C., FernándezAlemán J. L. (Aug. 2019). Reviewing Ensemble Classification Methods in Breast Cancer. *Computer Methods Programs Biomed*.

[6] MadhuKumari, Vijendra s. (2018). breast cancer prediction system” international conference on computational intelligence and data science. *Procedia Computer Science*.

[7] Abdar M., Makarenkov V. (2019). CWV-BANN-SVM Ensemble Learning Classifier for an Accurate Diagnosis of Breast Cancer. *Measurement*.

[8] Rajamohana S. P., Dharani A., Anushree P., Santhiya B., Umamaheswari K. (2019). Machine learning techniques for healthcare applications: early autism detection using ensemble approach and breast cancer prediction using SMO and IBK. *in Cognitive Social Mining Applications in Data Analytics and Forensics*.

[9] Togacar M., Ergen B. Deep learning approach for classification of breast cancer.

[10] Tiwari M., Bharuka R., Shah P., Lokare R. (2020). *‘Breast Cancer Prediction Using Deep Learning and Machine Learning Techniques*.

[11] Selvathi D., Poornila A. A. (2018). Deep learning techniques for breast cancer detection using medical image analysis. *in Biologically Rationalized Computing Techniques for Image Processing Applications*.

[12] Badr M., Al-Otaibi S., Alturki N., Abir T. (2022). Detection of heart arrhythmia on electrocardiogram using artificial neural networks. *Computational Intelligence and Neuroscience*.

[13] Hiba A., HajarMousannifb h., Al moatassime c., noeld t. Using machine learning algorithms for breast cancer risk prediction and diagnosis.

[14] Alghunaim, Al-Baity H. H. (2019). On the Scalability of Machine-Learning Algorithms for Breast Cancer Prediction in Big Data Context. *IEEE Access*.

[15] Hemeida a A. M., Salem Alkhalaf b, Mady c A., Mahmoud E. A., Hussein M. E., Ayman M., BahaEldin d. (June 2020). Implementation of nature-inspired optimization algorithms in some data mining tasks” Published by Elsevier B.V. on behalf of Faculty of Engineering. *Ain Shams University. Ain Shams Engineering Journal*.

[16] VenkateswaraRao L., Mary Gladence V., Lakshmi R. (2019). Research of Feature Selection Methods to Predict Breast Cancer. *International Journal of Recent Technology and Engineering*.

[17] Dhahri H., Al Maghayreh E., Mahmood A., Elkilani W., Faisal Nagi M. (2019). Automated breast cancer diagnosis based on machine learning algorithms. *Journal of Healthcare Engineering*.

[18] Walid C. (2018). Optimization of K-NN Algorithm by Clustering and Reliability Coefficients: Application to Breast-Cancer Diagnosis. *Elsevier Procedia Computer Science*.

[19] Huang H., Feng Xi’an, Zhou S. (2019). A new fruit fly optimization algorithm enhanced support vector machine for diagnosis of breast cancer based on high-level features. *BMC Bioinformatics*.

[20] SapiahBintiSakri N. B., Rashid A., Muhammad Z. (2018). Particle Swarm Optimization Feature Selection for Breast Cancer Recurrence Prediction. *Special Section on Big Data Learning and Discovery IEEE Access*.

[21] Hamed G., Marey M. A. E.-R., Amin S. E.-S., Tolba M. F. Deep learning in breast cancer detection and classification.

[22] Abdullah Hamad A., Thivagar M. L., Bader Alazzam M., Alassery F., Hajjej F., Shihab A. A. (2022). Applying dynamic systems to social media by using controlling stability. *Computational Intelligence and Neuroscience*.

[23] Bray F., Ferlay J., Soerjomataram I., Siegel R. L., Torre L. A., Jemal A. (2018). Global cancer statistics 2018: GLOBOCAN estimates of incidence and mortality worldwide for 36 cancers in 185 countries. *CA: A Cancer Journal for Clinicians*.

[24] Khalil S., Hatch L., Price C. R. (2019). Addressing Breast Cancer Screening Disparities Among Uninsured and Insured Patients: A Student-Run Free Clinic Initiative. *J Community Health*.

[25] Memis A., Ozdemir N., Parildar M., Ustun E. E., Erhan Y. (2000). ‘Mucinous (colloid) breast cancer: mammographic and US features with histologic correlation. *European Journal of Radiology*.

[26] Reddy A., Soni B., Reddy S. (2020). Breast Cancer Detection by Leveraging Machine Learning. *ICT Express*.

[27] Salod Z., Singh Y. (Dec. 2019). ‘Comparison of the performance of machine learning algorithms in breast cancer screening and detection: a protocol. *J. Public Health Res.*.

[28] Supriya M., Deepa A. J. (2019). A Novel Approach for Breast Cancer Prediction Using Optimized ANN Classifier Based on Big Data Environment” Health Care Management Science. *Springer, Science+Business Media, LLC, part of Springer Nature*.

[29] Siotos C., Naska A., Bello R. J. (2019). ‘‘Survival and Disease Recurrence Rates Among Breast Cancer Patients Following Mastectomy with or without Breast Reconstruction. *Plastic Reconstructive Surg*.

[30] Memon M. H., Li J. P., Haq A. U., Memon M. H., Zhou W. (2019). ‘Breast cancer detection in the IOT health environment using modified recursive feature selection. *Wireless Communications and Mobile Computing*.

[31] Kirola M., Memoria M., Dumka A., Tripathi A., Joshi K. (2022). A comprehensive review study on: optimized data mining, machine learning and deep learning techniques for breast cancer prediction in big data context. *Biomedical and Pharmacology Journal*.

[32] Kamel S. R., YaghoubZadeh R., Kheirabadi M. (2019). Improving the Performance of Support-Vector Machine by Selecting the Best Features by Gray Wolf Algorithm to Increase the Accuracy of Diagnosis of Breast Cancer. *J Big Data6*.

[33] Maray M., Alghamdi M., Alazzam M. B. (2022). Diagnosing cancer using IOT and machine learning methods. *Computational Intelligence and Neuroscience*.

[34] American Cancer Society (2018). *Global Cancer: Facts & Figures*.

[35] India against Cancer (2019).

[36] American Cancer Society (2019). *Breast Cancer Facts & Figures 2019-2020*.

[37] Mekha P., Teeyasuksaet N. Deep learning algorithms for predicting breast cancer based on tumor cells.

[38] Israni P. (2019). ‘Breast cancer diagnosis (BCD) model using machine learning. *‘‘ Int. J. Innov. Technol. Exploring Eng., Aug.*.

[39] Khourdifi, Bahaj M. Applying best machine learning algorithms for breast cancer prediction and classification.

[40] Lu Y., Li J.-Y., Su Y.-T., Liu A.-A. A review of breast cancer detection in medical images.

[41] Hou R., Mazurowski M. A., Grimm L. J. (2020). ‘Prediction of upstaged ductal carcinoma in situ using forced labeling and domain adaptation. *IEEE Transactions on Biomedical Engineering*.

[42] Bataineh A. A. (2019). ‘A comparative analysis of nonlinear machine learning algorithms for breast cancer detection. *International Journal of Machine Learning and Computing*.

[43] Keles M. K. (2019). Breast Cancer Prediction and Detection Using Data Mining Classification Algorithms: A Comparative Study. *Tehnički Vjesnik*.

